The article "In-silico modelling studies of 5-benzyl-4-thiazolinone derivatives as influenza neuraminidase inhibitors via 2D-QSAR, 3D-QSAR, molecular docking, and ADMET predictions" was retracted in 2023. Reasons: no approval from a third party; copyright claims.

# In-silico modelling studies of 5-benzyl-4-thiazolinone derivatives as influenza neuraminidase inhibitors via 2D-QSAR, 3D-QSAR, molecular docking, and ADMET predictions

**DOI:** 10.1016/j.heliyon.2022.e10101

**Published:** 2022-08-08

**Authors:** Mustapha Abdullahi, Adamu Uzairu, Gideon Adamu Shallangwa, Paul Andrew Mamza, Muhammad Tukur Ibrahim

**Affiliations:** a Faculty of Physical Sciences, Department of Chemistry, Ahmadu Bello University, P.M.B. 1044, Zaria, Kaduna State, Nigeria; b Faculty of Sciences, Department of Pure and Applied Chemistry, Kaduna State University, Tafawa Balewa Way, Kaduna, Nigeria

**Keywords:** Modelling, Binding energy, Influenza, Neuraminidase, Residual interaction

## Abstract

Influenza virus disease is one of the most infectious diseases responsible for many human deaths, and the high mutability of the virus causes drug resistance effects in recent times. As such, it became necessary to explore more inhibitors that could avert future influenza pandemics. The present research utilized some in-silico modelling concepts such as 2D-QSAR, 3D-QSAR, molecular docking simulation, and ADMET predictions on some 5-benzyl-4-thiazolinone derivatives as influenza neuraminidase (NA) inhibitors. The 2D-QSAR modelling results revealed GFA-MLR (${\text{R}}_{\text{train}}^{2}$ =0.8414, Q^2^ = 0.7680) and GFA-ANN (${\text{R}}_{\text{train ​}}^{2}$ =0.8754, Q^2^ = 0.8753) models with the most relevant descriptors (MATS3i, SpMax5_Bhe, minsOH and VE3_D) for predicting the inhibitory activities of the molecules which has passed the global criteria of accepting QSAR models. The results of the 3D-QSAR modelling results showed that CoMFA_ES (${\text{R}}_{\text{train ​}}^{2}$ =0.9030, Q^2^ = 0.5390) and CoMSIA_EA (${\text{R}}_{\text{train}}^{2}$ =0.880, Q^2^ = 0.547) models are having good predicting ability among other developed models. The molecules were virtually screened via molecular docking simulation with the active site of NA protein receptor (pH1N1) which confirms their resilient potency when compared with zanamivir standard drug. Molecule 11 as the most potent molecule formed more H-bond interactions with the key residues such as TRP178, ARG152, ARG292, ARG371, and TYR406 that triggered the catalytic reactions for NA inhibition. Furthermore, six (6) molecules (9, 10, 11, 17, 22, and 31) with relatively high inhibitory activities and docking scores were identified as the possible leads for in-silico exploration of novel NA inhibitors. The drug-likeness and ADMET predictions of the lead molecules revealed non-violation of Lipinski’s rule and good pharmacokinetic profiles respectively, which are important guidelines for rational drug design. Hence, the outcome of this study overlaid a solid foundation for the in-silico design and exploration of novel NA inhibitors with improved potency.

## 1 Introduction

Influenza virus disease remains one of the major health menaces affecting humans because of its high mortality and morbidity rates in recent times even with the devastating Covid-19 pandemic (Akhtar et al., 2021). The World Health Organization (WHO) reported about 2–5 million cases of severe illness caused by the ravaging seasonal influenza virus epidemic which resulted in over 500,000 deaths globally (Korsten et al., 2021). These flu epidemics cause severe respiratory infections in children, adults, the elderly, and people with underlying health conditions (Aleebrahim-Dehkordi et al., 2022). Influenza virus neuraminidase (NA) is an enzyme that catalyzes the obliteration of terminal sialic acid residues (sialidase) which aids in liberating new virions formed from the infected cells and circulating to infect the neighboring cells (Abed et al., 2016). As such, the NA inhibition can defend the host from being infected and prevent its proliferation (Avila et al., 2020). Due to the highly preserved active site structure of neuraminidase (Adams et al., 2019), it has become an attractive molecular target for the exploration and development of novel anti-influenza inhibitors. Nowadays, zanamivir (Relenza™), oseltamivir (Tamiflu™), laninamivir octanoate (Inavir™), and peramivir (Rapivab™) are the four (4) approved neuraminidase inhibitors for influenza treatment (Hayden et al., 2022). Although, there is a lot of concern for the advent of drug resistance effects resulting from the high variability of the influenza virus (Abed et al., 2016). Hence, there is a need to explore more anti-influenza drugs that have more potent efficiency and binding modes with safer side effects than the currently available drugs. The compounds of thiazolidin-4-onealso known as 4-thiazolinones were reported to have an extensive biological activity range such as anti-fungal, anti-inflammatory, anti-cancer, anti-bacterial, and anti-viral amongst others (Xiao et al., 2021). The trial and error approach applied in the development of new drugs has been seen to be very tedious, costly, and time-consuming (Abdullahi et al., 2021). Hence, the validation of reported anti-influenza agents with the aim of improve them remains an area of high research interest. The application of some in-silico modelling concepts such as quantitative structure-activity relationship (2D-QSAR and 3D-QSAR), molecular docking, and ADMET studies can save time of filteringhits-to-leads, and reduce the cost of synthesizing newly potent drugs (Al-Attraqchi and Venugopala, 2020). In this study, the in-silico modelling concepts such as 2D-QSAR, 3D-QSAR, molecular docking, and ADMET predictions were applied to identify probable lead candidates for the future in-silico design of new anti-influenza agents with improved bioactivities. The 2D-QSAR and 3D-QSAR modelling studies were carried out on 48 compounds of 5-benzyl-4-thiazolinone to predict their anti-influenza activity using some computed structural features of the compounds in numerical values (molecular descriptors). The 2D-QSAR model was initially constructed based on genetic function approximation-multi-linear regression (GFA-MLR) and the subsequent artificial neural regression (GFA-ANN) analysis. The 3D-QSAR models were constructed based on the comparative molecular field analysis (CoMFA) and comparative similarity indices analysis (CoMSIA) methods for the activity prediction of the molecules. The 48 molecules were virtually screened with the NA protein target to identify possible lead candidates based on their docking scores and residual interactions via molecular docking studies. Finally, the physicochemical properties of the molecules were generated to study their drug-likeness and pharmacokinetic profiles.

## 2 Methodology

### 2.1 Data set collection and biological activities (pIC_50_)

A data set containing 48 molecules of 5-benzyl-4-thiazolinone derivatives as inhibitors of influenza (H1N1) neuraminidase (NA) were obtained from the previously published work of Xiao et al. (2021). The reported NA inhibitory activities of the molecules evaluated in IC_50_ (μM) were further transformed to a logarithmic scale (pIC_50_ = −log IC_50_ × 10^−6^) to eliminate data skewness for the QSAR studies (Abdullahi et al., 2020b). Thirty-five (35) molecules were used as a training set while the remaining 13 molecules were used as the test set as presented in Table 1.

**Table 1:** Data set of 5-benyl-4-thiazolinone derivatives along with their inhibitory activities.


Sr No.	R^1^	R^2^	R	IC_50_ (μM)	pIC_50_
1	CO_2_CH_2_CH_3_	CH_3_	2-OH	28.78	4.5409
2	CO_2_CH_2_CH_3_	CH_3_	3-OH	43.57	4.3608
3	CO_2_CH_2_CH_3_	CH_3_	3-OCH_3_	73.11	4.1360
4	CO_2_CH_2_CH_3_	CH_3_	3-F	64.38	4.1912
5	CO_2_CH_2_CH_3_	CH_3_	3-Cl	78.72	4.1039
6	CO_2_CH_2_CH_3_	CH_3_	4-CO_2_H	36.46	4.4381
7	CO_2_CH_2_CH_3_	CH_3_	4-CO_2_Me	94.02	4.0267
∗8	CO_2_CH_2_CH_3_	CH_3_	4-NHAc	44.11	4.3554
9	CO_2_CH_2_CH_3_	CH_3_	4-OH	16.33	4.7870
10	CO_2_CH_2_CH_3_	CH_3_	2-OH-3-OCH_3_	19.21	4.7164
11	CO_2_CH_2_CH_3_	CH_3_	3-OCH_3_-4-OH	13.06	4.8840
12	CO_2_CH_2_CH_3_	CH_3_	2,4-(OH)_2_	28.31	4.5480
13	CO_2_CH_2_CH_3_	CH_3_	3,4-(OH)_2_	27.11	4.5668
14	CO_2_CH_2_CH_3_	CH_3_	2-OH-3,5-di NO_2_	39.86	4.3994
∗15	CO_2_H	CH_3_	3-OCH_3_-4-OH	32.47	4.4885
16	CO_2_CH_3_	CH_3_	3-OCH_3_-4-OH	30.39	4.5172
17	CO_2_*t*-Bu	CH_3_	3-OCH_3_-4-OH	27.53	4.5601
18	CO_2_ CH_3_	*i*-Pr	4-OH	19.21	4.7164
∗19	CO_2_ CH_3_	*i*-Pr	2-OH-3-OCH_3_	28.90	4.5391
20	CO_2_ CH_3_	*i*-Pr	3,4-(OH)_2_	21.81	4.6613
21	CO_2_CH_3_	*i*-Pr	3-OCH_3_-4-OH	22.98	4.6386
22	CO_2_CH_3_	*i*-Pr	3,5-(OCH_3_)_2_-4-OH	28.67	4.5425
23	CO_2_CH_3_	*n*-Pr	3-OCH_3_-4-OH	30.43	4.5166
24	H	CH_2_CO_2_CH_2_CH_3_	3-NO_2_	46.00	4.3372
25	H	CH_2_CO_2_CH_2_CH_3_	3-NH_2_	35.76	4.4466
26	H	CH_2_CO_2_CH_2_CH_3_	4-CO_2_H	34.71	4.4595
∗27	H	CH_2_CO_2_CH_2_CH_3_	4-OH	27.69	4.5576
28	H	CH_2_CO_2_CH_2_CH_3_	2-OH-3-OCH_3_	33.90	4.4698
29	H	CH_2_CO_2_CH_2_CH_3_	3-OH-4-OCH_3_	28.80	4.5406
∗30	H	CH_2_CO_2_CH_2_CH_3_	3-OCH_3_-4-OH	28.04	4.5522
∗31	CH_3_	CH_2_CO_2_CH_2_CH_3_	3-OCH_3_-4-OH	20.30	4.6925
32	Ac	CH_3_	3-NO_2_	70.54	4.1515
33	Ac	CH_3_	3-OH	19.09	4.7191
∗34	Ac	CH_3_	4-CO_2_H	31.75	4.4982
35	Ac	CH_3_	4-OH	20.53	4.6876
36	Ac	CH_3_	3-OH-4-OCH_3_	18.28	4.7380
37	Ac	CH_3_	3-OCH_3_-4-OH	26.11	4.5831
∗38	Ac	CH_3_	3,4-OCH_2_O	42.28	4.3738
∗39	Ac	CH_3_	3,4-(OH)_2_	25.30	4.5968
40	NO_2_	*t*-Bu	2-CO_2_H	33.02	4.4812
41	NO_2_	*t*-Bu	2-OH	35.36	4.4514
42	NO_2_	*t*-Bu	3-NO_2_	48.24	4.3165
43	NO_2_	*t*-Bu	3-OCH_3_	44.18	4.3547
44	NO_2_	*t*-Bu	3-F	32.08	4.4937
45	NO_2_	*t*-Bu	4-NHAc	75.78	4.1204
46	NO_2_	*t*-Bu	4-OH	38.82	4.4109
∗47	NO_2_	*t*-Bu	2-OH-3-OCH_3_	55.03	4.2594
∗48	NO_2_	*t*-Bu	3-OCH_3_-4-OH	35.21	4.4533

∗ superscript = test set.

### 2.2 2D-QSAR studies

#### 2.2.1 Generation of 2D descriptors

The chemical structures of the 48 molecules in the dataset were accurately drawn using ChemDraw software, then exported to Spartan 14 for initial geometry minimization using molecular mechanics force fields (MMFF). The minimized structures were further optimized at the DFT level (B3LYP/631G∗∗) to determine their most stable conformation using Spartan 14 (Abdullahi et al., 2020a). PaDEL Descriptor tool was then used to calculate about 2000 molecular descriptors from the optimized structures. These molecular descriptors are computed based on their steric potentials, electronic properties, potential hydrogen bonds of path length, relative ionization, and hydrophobicity which are functions of bioactivities (Ahamad et al., 2019).

#### 2.2.2 Data pretreatment and division

The calculated molecular descriptors were pretreated to generate a robust model by removing highly inter-correlated and redundant values (Apablaza et al., 2017). Furthermore, the pretreated descriptors were divided into training (model development set) and test set (model validation set) using Kennard and Stone’s algorithm.

#### 2.2.3 Construction of the 2D-QSAR models

The construction of the QSAR model was established by employing the Material Studio software version 8.0. The Genetic Function Approximation (GFA) was used for the feature selection of the pretreated descriptors in the training set for model development (Abdullahi et al., 2020a), and Friedman Lack-of-Fit (LOF) was selected as the functionality while the scaled LOF smoothness parameter was set at the default of 0.5. The population sample was set to 10,000 at 1000 maximum generations and the number of top equations return was set to 1 (Umar et al., 2019). The descriptor matrix of the best-built model was initially subjected to the *Y-Randomization test* as a measure to attest to the quality of the model before being exported to Molegro Data Modeller (MDM) software for the development of the MLR and ANN models (Poleboyina et al., 2022). The MLR model assumes that the dependent variable (*y*) is a linear function of the independent variables (*x*_*i*_), as shown in Eq. (1).

(1) $$y=c_{0}+\overset{n}{\underset{i=1}{\sum }}c_{i}x_{i}$$

Where *y* represents the inhibitory activity (pIC_50_), *x*_*i*_ represents the molecular descriptors, $c_{i}$ is the regression coefficient in the linear model, and $c_{0}$ is the intercept of the equation (constant). On the other hand, artificial neural networks are simulated by the biological neural networks of the real world. The artificial systems of the neural networks are simulating the function of the human brain which has shown good performance on classification and regression problems (Darnag et al., 2017). These networks are developed by representing each independent variable as a neuron in the input layer, and connections are formed to other neurons in the next layer (hidden layer). Each of the connections is multiplied by the neuron output layer by a weighted score (Bouakkadia et al., 2021). Hence, the output layer (pIC_50_) is computed by applying a sigmoid function and summing all inputs as shown in Eqs. (2) and (3) respectively.

(2) sigmoid ​(x)=1(1+e−x)

(3) $$\text{output ​}\left({\text{pIC}}_{50}\right)=\text{sigmoid ​}\left(\sum \text{input}\right)$$

#### 2.2.4 Model applicability domain (AD)

The model applicability domain is the theoretical chemical space of the compounds defined by the descriptors and the modeled activity in which the acceptable 2D-QSAR model can make reliable predictions (Abdullahi et al., 2020b). Thus, the technique helps in detecting the structural and response outliers in the training and test set respectively. Furthermore, the leverage approach was utilized to assess the chemical space of the best QSAR model, and the plot of standardized residuals against leverage values (h) also known as the Williams plot was used to assess the chemical space (Ibrahim et al., 2020). As such, compounds with leverage scores less than the threshold (h < h∗) and standardized residual scores within ±3.0σ (standard deviation unit) are set to have fallen in the model's chemical space or applicability domain. The warning leverage (h∗) is calculated using Eq. (4):

(4) $$h^{*}=3\frac{\left(d+1\right)}{\text{N}}$$

Where d is the number of descriptors in the model and N is the number of compounds used as the training set.

### 2.3 3D-QSAR studies

#### 2.3.1 Molecular minimization and alignment

The optimized structures were minimized with Gasteiger-Huckel atomic charges of Tripos force field based on Powell conjugate gradient algorithm method at convergence criteria of 0.05 kcal/(mol Å) and 1000 maximum iterations to determine their steady conformation using Sybyl-X 2.1.1 program (Abdizadeh et al., 2017). The molecular alignment of a database is one of the most crucial steps for building a reliable and predictive 3D-QSAR model. Distill rigid alignment method was used to align the molecules in the database to the most potent compound in the dataset **(molecule no. 11**) as the template with the common core or backbone produced as shown in Figure 1.

**Figure 1:** 3D-QSAR optimized structures, (A) distill rigid common core, (B) optimized structure of molecule 11, (C) alignment and superposition of the 5-benzyl-4-thiazolinone derivatives (Strick model).

#### 2.3.2 Development of 3D QSAR models

The CoMFA and CoMSIA methods were used to generate the 3D-QSAR models of the NA inhibitors using SYBYL-X 2.1.1 software (Tripos Inc) to explain the relationship between the inhibitory activity (pIC_50_) as the dependent variable and the 3D structure of molecules (Vishwakarma and Bhatt, 2021). The descriptor parameters of the built CoMFA model were electrostatic (E) and steric (S) energy values at a point in space surrounding the molecules while the CoMSIA model was built with more additional field descriptors such as steric(S), electrostatic (E), hydrophobic (H), hydrogen bond donor (HBD) field, hydrogen bond acceptor (HBA) for both training and test set (Goudzal et al., 2022).

### 2.4 Internal and external validation of the 2D and 3D QSAR models

For the 2D-QSAR modelling, the GFA-MLR model building protocol of Material Studio was initially used for the feature selection of the best descriptors matrix (independent variable) to predict the dependent variable (pIC_50_) (Abdullahi et al., 2020a). Subsequently, molegro data modeller (MDM) was used to generate statistical validation metrics for the 2D-QSAR model based on MLR and ANN regression analysis (Vyas and Georrge, 2015). The prediction capability of the 2D-QSAR models generated was assessed using internal and external validation parameters such as Pearson correlation coefficient (R), adjusted R^2^, Spearman’s rank correlation coefficient (ρ), cross-validated regression coefficient (Q^2^), root mean square error (RMSE), predicted coefficient of determination for the test set $\;\left({\text{R}}_{\text{Pred}}^{2}\right)$, regression coefficients for the training and test set (${\text{R}}_{\text{train ​}}^{2}\text{and}\;{\text{R}}_{\text{test}}^{2})$, and coefficient of determination of Y-randomization $\left(CR_{p}^{2}\right)$ whose calculation formulas are shown in Eqs. (5), (6), (7), (8), (9), (10), (11), and (12).

(5) $${\text{R}}_{\text{train ​}}^{2}or\;{\text{R}}_{\text{test}}^{2}=\frac{{\left[\sum \left\{\left({\text{Y}}_{\text{actual}}-{\text{Y}}_{\text{mean}}\right)\left({\text{Y}}_{\text{predict}}-{\bar{\text{Y}}}_{\text{pred}}\right)\right\}\right]}^{2}}{\sum {\left({\text{Y}}_{\text{actual}}-{\text{Y}}_{\text{mean}}\right)}^{2}\sum {\left({\text{Y}}_{\text{predict}}-{\bar{\text{Y}}}_{\text{pred}}\right)}^{2}}$$

(6) $${\text{Adjusted ​R}}^{2}=1-\left(1-{\text{R}}^{2}\right)\frac{\text{N}-1}{\text{N}-\text{p}-1}$$

(7) $$\text{ρ}=1-\frac{6\sum_{\text{i}=1}^{\text{N}}{\text{d}}_{\text{i}}^{2}}{\text{N}\left({\text{N}}^{2}-1\right)}$$

(8) $$Q^{2}=\;1.0\;–\frac{\sum_{Y}{\left({\text{Y}}_{\text{predict}}-{\text{ ​Y}}_{\text{actual}}\right)}^{2}}{\sum_{Y}{\left({\text{Y}}_{\text{actual}}-{\text{ ​Y}}_{\text{mean}}\right)}^{2}}$$

(9) $$SEE=\;\sqrt{\frac{{\left({\text{Y}}_{\text{predict}}-{\text{ ​Y}}_{\text{actual}}\right)}^{2}}{n-c-1}}$$

(10) $$R_{pred}^{2}=1.0\;-\;\frac{\sum {\left({\text{Y}}_{{\left(\text{test}\right)}_{\text{actual}}}-{\text{ ​Y}}_{{\left(\text{test}\right)}_{\text{predict}}}\right)}^{2}}{\sum {\left({\text{Y}}_{{\left(\text{test}\right)}_{\text{actual}}}-{\text{ ​Y}}_{{\left(\text{training}\right)}_{\text{mean}}}\right)}^{2}}$$

(11) $$CR_{p}^{2}={\text{ ​R}}^{2}\times {\left({\text{R}}^{2}-{\left(\bar{R_{r}}\right)}^{2}\right)}^{0.5}$$

(12) $$\text{RMSE}=\sqrt{\frac{\sum_{\text{i}=1}^{\text{N}}{\left({\text{Y}}_{\text{predict}}-{\text{ ​Y}}_{\text{actual}}\right)}^{2}}{\text{N}}}$$

The correlation coefficient squared (R^2^) is often used to describe relationships between two variables whose range of value is between 0 and 1. N is the number of compounds in the training set as data points and p is the number of descriptors in the built model. d_i_ is the difference between the ranks of corresponding values predicted and actual responses. ${\text{Y}}_{\text{predict}}$ is the predicted response activity, ${\text{Y}}_{\text{actual}}$ is the actual response activity, ${\text{Y}}_{\text{mean}}$ is the mean value of the actual response activity, and the numerator is PRESS, ${\text{Y}}_{{\left(\text{test}\right)}_{\text{actual}}}$ is the actual response activity of the test set, ${\text{Y}}_{{\left(\text{test}\right)}_{\text{predict}}}$ is the predicted response activity of the test set, ${\text{Y}}_{{\left(\text{training}\right)}_{\text{mean}}}$ is the actual mean response activity of the training set, *c* is the number of components, and $\bar{R_{r}}$ is the average R of random models (Roy et al., 2016; Roy et al., 2015a, b).

On the other hand, the 3D-QSAR models were constructed by correlating the latent components from the set of available CoMFA and CoMSIA descriptors (independent variable) with the inhibitory activities of the molecules through the partial least squares (PLS) regression analysis (Aouidate et al., 2018). The predictive performance of both models was assessed based on some prominent internal and external validation metrics such as cross-validated (Q^2^), cross-validated standard error of estimate (SEE), regression coefficients for the training and test set (${\text{R}}_{\text{train}}^{2}\;\&\;{\text{R}}_{\text{test}}^{2})$, and predicted coefficient of determination for the test set $\;\left({\text{R}}_{\text{Pred}}^{2}\right)$ (Tropsha, 2010; Vucicevic et al., 2019). A concise workflow diagram displaying the general overview processes adopted in this study for the construction of the 2D and 3D-QSAR models was shown in Figure 2.

**Figure 2:** Workflow diagram of constructing 2D and 3D-QSAR models.

### 2.5 Molecular docking investigation

A molecular docking investigation was carried out to further predict the potential bindings between neuraminidase protein and the 48 molecules of 5-benzyl-4-thiazolinone derivatives using molecular operating environment (MOE) V2015.10 software. The crystal structure of the 2009 influenza pandemic H1N1 (pH1N1) neuraminidase complexed with zanamivir (PDB: 3TI5) was selected as the template protein while the co-crystalized ligand was used as the reference drug (Vavricka et al., 2011).

#### 2.5.1 Energy minimization and the docking protocol

The 5-benzyl-4-thiazolinone molecules were initially imported to the MOE builder interface for energy minimization and conformational searching until an RMS distance of 0.1 Å and RMSD gradient of 0.01 kcal/mol were computed for each molecule using Amber12: ET force field. The database of the molecules was later saved for the docking protocol (Ahmed et al., 2021). The pH1N1 neuraminidase was also minimized by fixing all hydrogen atoms, lone pairs, and partial charges accordingly. To increase the docking accuracy, the co-crystalized ligand was initially re-docked to analyze the ligand-active pocket interactions, and the RMSD scores were calculated between the docked poses and the co-crystalized ligand. The MOE program was adjusted to the triangle matcher method based on the London dG scoring function for placement selection and induced fit with GBVI/WSA dG scoring function for refinement before the docking starts (Shakour et al., 2021). The database of ligands in MDB file docked (zanamivir and the thiazolinones) were then imported, and the docking simulation was executed for screening based on their binding scores.

### 2.6 Drug likeness and ADMET prediction studies

The preliminary estimation of physicochemical, drug-likeness and pharmacokinetic parameters of potential drug candidates is crucial, especially at the initial stage of the drug discovery process which helps in rolling out unfavourable effects of the candidates (Aziz et al., 2022). The pharmacokinetic parameters are based on desirable adsorption, distribution, metabolism, excretion, and toxicity (ADMET) of the query drug when administered into the body (Ibrahim et al., 2020). An efficient and accurate ADMETlab 2.0 webserver (https://admetmesh.scbdd.com/) was utilized to predict numerous physicochemical, drug-likeness, pharmacokinetic, and toxicity parameters of molecules in the study (Babalola et al., 2022; Kar et al., 2022). In addition, the drug-likeness of the 5-benzyl-4-thiazolinones (48 molecules) was assessed based on Lipinski, Ghose, Veber, Egan, and Muegge rules using the SwissADME online webserver at http://www.swissadme.ch/index.php.

## 3 Results and discussion

### 3.1 2D-QSAR models validation results

The 2D-QSAR modelling approach was successfully carried out on the 5-benzyl-4-thiazolinone derivatives as novel inhibitors against the H1N1 neuraminidase target. The built 2D-QSAR model in this study was used to predict anti-influenza response activities with the influence of some robust and statistically significant descriptors (Ibrahim et al., 2020). As mentioned earlier, the GFA model building protocol of Material Studio software was used for the selection of the best model descriptors. Subsequently, a 2D-QSAR model was successfully derived using MDM software based on the MLR and the subsequent ANN regression modelling with the five (5) best descriptors whose model internal and external validation metrics were shown in Tables 2 and 3 respectively.

**Table 2:** Internal validation of the 2D-QSAR models.

Internal validation metrics	GFA- MLR	GFA-ANN (5-3-1)	Threshold	Comment	Reference
Lack of fit (LOF)	0.0341	-			
Pearson Correlation (R)	0.9173	0.9360	R > 0.6	Passed	(Tropsha, 2010)
Pearson Correlation squared (${\text{R}}_{\text{train ​}}^{2}$)	0.8414	0.8754	R^2^_train_ > 0.6	Passed	(Tropsha, 2010)
Adjusted r^2^	0.8140	-	R^2^_adj_ > 0.6	Passed	(Tropsha, 2010)
Spearman Rank Correlation (ρ)	0.9112	0.9356	ρ > 0.6	Passed	
Root Mean Squared Deviation (RMSE)	0.0802	0.0711	Low	Passed	
Cross Validated Squared (Q^2^)	0.7680	0.8753	Q^2^ > 0.6	Passed	(Tropsha, 2010)
Y-randomization ($cR_{p}^{2})$	0.7581	-	$cR_{p}^{2}$ >0.6	Passed	(Roy et al., 2016)

**Table 3:** External validation parameters of the 2D-QSAR models.

External validation metrics	GFA- MLR Model	GFA-ANN (5-3-1)	Threshold	Comment	Reference
Pearson Correlation squared (${\text{R}}_{\text{test}}^{2}$)	0.6975	0.7003	R^2^_test_ > 0.6	Passed	(Tropsha, 2010)
$R_{pred}^{2}$	0.6034	0.5899	$R_{pred}^{2}$ >0.5	Passed	
Δ ${\bar{R}}_{m}^{2}$ (test)	0.0842	-	<0.5	Passed	
$r_{0}^{2}$	0.6585	-	>0.5	Passed	
RMSEP	0.0863	0.0827	-	-	
r'^2^_0_	0.6797	-	>0.5	Passed	(Tropsha, 2010)
(r^2^-r_0_^2^)/r^2^	0.0558	-	(r^2^-r_0_^2^)/r^2^ < 0.1	Passed	
K	0.9927	-	0.85 < k < 1.15	Passed	
(r^2^- r'^2^_0_)/r^2^	0.0254	-	(r^2^- r'^2^_0_)/r^2^ < 0.1	Passed	
k’	1.0069	-	0.85 < k’ < 1.15	Passed	
$\left|r_{0}^{2}-\text{r}{\text{′}}_{0}\right|$	0.0211	-	$\left|r_{0}^{2}-\text{r}{\text{′}}_{0}\right|$ <0.3	Passed	

The proposed 2D QSAR model equation was given below as Eq. (13);

(13) $$\text{Inhibitory ​activity ​}\left({\text{pIC}}_{50}\right)=-0.665892\text{ ​∗ ​ATSC}6\text{c ​}+0.584588\text{ ​∗ ​MATS}3\text{i ​}-1.24459\text{ ​∗ ​SpMax}5\_\text{Bhe ​}+0.0236721\text{ ​∗ ​minsOH ​}+0.0326316\text{ ​∗ ​VE}3\_\text{D ​}+8.75957$$

The prediction quality of the GFA-MLR model was assessed using the validation metrics such as correlation coefficient (R^2^) of 0.8414, adjusted R^2^ of 0.8140, and cross-validation correlation coefficient (Q^2^) of 0.7680 for the training set, ${\text{R}}_{\text{test}}^{2}$ of 0.6975, and ${\text{R}}_{\text{pred}}^{2}$ of 0.6034 accordingly. The Y-Randomization test was ascertained by randomly scrambling of the inhibitory activity (*y*) and the model descriptors of the training set are kept constant which resulted in the construction of random models (Roy et al., 2016). The 50 random models were generated with low R^2^ and Q^2^ scores which attested that the original model is robust and not constructed by chance (Roy et al., 2015b). The coefficient of determination for the Y-randomization test ($cR_{p}^{2})$ was computed as 0.7581 (≥0.5) which confirmed the reliability of the model generated as shown in Table 4. Hence, the validation parameters generated in this study were within the acceptable threshold parameters as reported in the previous QSAR researches (Tropsha, 2010). Using the same five (5) subset descriptors as the input layer and a single hidden layer with 3 neurons (Figure 3), a GFA-ANN (5-3-1) regression model was constructed to examine the best non-linear relationship between the response activities and the model variables. The predicted inhibitory activity values of the molecules constitute a single output layer which is computed using a sigmoid transfer function. The model was built at default parameter set up in the MDM tool (max epochs = 1000, momentum = 0.2, general/output layer learning rate = 0.3). The result indicates an improved statistical parameter of validation such as R^2^ (training set) of 0.8754, cross-validation (Q^2^) of 0.8753, RMSE of 0.0711, ${\text{R}}_{\text{test}}^{2}$ of 0.7003, and ${\text{R}}_{\text{pred}}^{2}$ of 0.5899 as shown in Tables 2 and 3 accordingly.

**Table 4:** Y-randomization test of the model descriptors.

MODEL	R	R^2^	Q^2^ (LOO)	MODEL	R	R^2^	Q^2^ (LOO)
Original	0.9173	0.8414	0.7681	Original	0.9173	0.8414	0.7681
Random 1	0.3574	0.1278	-0.3666	Random 26	0.1883	0.0355	-0.4099
Random 2	0.4594	0.2110	-0.2035	Random 27	0.4261	0.1816	-0.2759
Random 3	0.6423	0.4125	0.1551	Random 28	0.3670	0.1347	-0.2425
Random 4	0.4056	0.1645	-0.2584	Random 29	0.2001	0.0400	-0.4476
Random 5	0.3451	0.1191	-0.3870	Random 30	0.5056	0.2556	-0.0475
Random 6	0.4313	0.1860	-0.1520	Random 31	0.5078	0.2579	-0.0803
Random 7	0.4283	0.1834	-0.1529	Random 32	0.3403	0.1158	-0.3843
Random 8	0.2939	0.0864	-0.2523	Random 33	0.3982	0.1586	-0.2892
Random 9	0.4702	0.2211	-0.2299	Random 34	0.4203	0.1767	-0.2389
Random 10	0.4601	0.2116	-0.1496	Random 35	0.2010	0.0404	-0.4155
Random 11	0.5903	0.3485	0.0092	Random 36	0.1324	0.0175	-0.4710
Random 12	0.4882	0.2383	-0.1971	Random 37	0.3296	0.1087	-0.2136
Random 13	0.2064	0.0426	-0.4425	Random 38	0.5965	0.3558	0.0670
Random 14	0.4616	0.2131	-0.0565	Random 39	0.4398	0.1934	-0.1688
Random 15	0.3612	0.1305	-0.2809	Random 40	0.2732	0.0746	-0.2944
Random 16	0.2242	0.0502	-0.4404	Random 41	0.5819	0.3386	0.0801
Random 17	0.4770	0.2275	-0.1251	Random 42	0.4008	0.1607	-0.2296
Random 18	0.4521	0.2044	-0.1910	Random 43	0.3549	0.1260	-0.3604
Random 19	0.5014	0.2514	-0.0418	Random 44	0.3377	0.1141	-0.2984
Random 20	0.4896	0.2397	-0.1612	Random 45	0.3193	0.1019	-0.3648
Random 21	0.4392	0.1929	-0.1599	Random 46	0.4605	0.2120	-0.1540
Random 22	0.4078	0.1663	-0.1980	Random 47	0.4489	0.2015	-0.1382
Random 23	0.4914	0.2414	-0.1107	Random 48	0.4655	0.2167	-0.1767
Random 24	0.3306	0.1093	-0.2728	Random 49	0.5281	0.2789	-0.0766
Random 25	0.2410	0.0581	-0.4051	Random 50	0.2152	0.0463	-0.3323

**Random Models Parameters**	
Average R	0.40808
Average R^2^	0.18476
Average Q^2^	-0.20129
CRp^2^	0.75814

**Figure 3:** Schematic representation of the GFA-ANN (5-3-1) architecture.

The description name of the model descriptors coded as, ATSC6c, MATS3i, SpMax5_Bhe, minsOH, and VE3_D, along with their computed numerical scores were shown in Tables 5 and 6, while the correlation statistical parameters such as correlation coefficient, VIF, and mean effect of the descriptors were shown in Table 7. The Pearson correlation of less than 0.5 signifies that there is no inter-correlation among each descriptor pair. The variance inflation factor (VIF) was calculated using Eq. (14), where R^2^ is the Pearson correlation coefficient.

(14) VIF=1(1−R2)

**Table 5:** Description of the model descriptors.

Descriptor Class	Description	Descriptor code
2D	Centered Broto-Moreau autocorrelation - lag 6/weighted by charges	ATSC6c
2D	Moran autocorrelation - lag 3/weighted by first ionization potential	MATS3i
2D	Largest absolute eigenvalue of Burden modified matrix - n 5/weighted by relative Sanderson electronegativities	SpMax5_Bhe
2D	Minimum atom-type E-State: –OH	minsOH
2D	Logarithmic coefficient sum of the last eigenvector from Barysz matrix/weighted by atomic number	VE3_D

**Table 6:** Computed model descriptors and activity predictions by the 2D-QSAR models.

CompID	ATSC6c	MATS3i	SpMax5_Bhe	minsOH	VE3_D	Response(Y)	MLR-Train (5D)	ANN-Train (5-3-1)
Training set								
5	−0.0375	−0.0729	3.1193	0.0000	−19.7602	4.1039	4.2150	4.1626
6	0.1276	−0.1003	3.2823	8.9507	−8.3948	4.4382	4.4688	4.4815
7	0.1126	−0.1202	3.3476	0.0000	−8.2125	4.0268	4.1800	4.1615
9	−0.0195	−0.0890	3.1306	9.3365	−9.2794	4.7870	4.7424	4.7388
10	0.1387	−0.0847	3.1767	10.2174	−8.1017	4.7165	4.6416	4.6236
11	−0.0992	−0.0844	3.1816	9.6898	−11.1457	4.8841	4.6821	4.7051
12	0.2074	−0.1049	3.1318	9.3573	−10.1519	4.5481	4.5526	4.5588
13	−0.0963	−0.1045	3.1378	9.3735	−14.7701	4.5669	4.5972	4.6398
14	0.1685	−0.1388	3.4118	10.1547	−5.7038	4.3995	4.3742	4.3902
16	−0.1046	−0.1982	3.1706	9.6740	−13.3883	4.5173	4.5594	4.5728
17	−0.0880	−0.1740	3.1914	9.7184	−15.0979	4.5602	4.4819	4.4957
18	−0.1676	−0.2553	3.2754	9.3597	−5.7734	4.7165	4.6786	4.6438
20	−0.2444	−0.2641	3.2772	9.3967	−6.9513	4.6613	4.6848	4.6607
21	−0.2473	−0.2407	3.2813	9.7129	−7.8260	4.6386	4.6742	4.6579
22	−0.4464	−0.2245	3.2835	10.0662	−16.1842	4.5426	4.5491	4.5668
1	0.2182	−0.0894	3.1147	9.8641	−9.5154	4.5409	4.6085	4.5991
23	−0.1308	−0.1320	3.3020	9.7280	−9.3598	4.5167	4.5848	4.5956
24	0.1818	−0.0606	3.3044	0.0000	−6.0181	4.3372	4.2941	4.3096
25	0.2493	−0.0600	3.1834	0.0000	−5.8583	4.4466	4.4052	4.4783
26	0.3789	−0.0534	3.2819	8.9452	−8.2546	4.4595	4.3338	4.3740
28	0.3899	−0.0423	3.1937	10.2073	−5.1919	4.4698	4.5726	4.5466
29	0.2152	−0.0420	3.2066	9.8852	−6.5408	4.5406	4.6214	4.6072
32	−0.0085	−0.1288	3.2748	0.0000	−13.8889	4.1516	4.1609	4.1145
33	0.0245	−0.1209	3.0892	9.5121	−10.5836	4.7192	4.7076	4.7026
35	0.0416	−0.1209	3.0999	9.3117	−7.5760	4.6876	4.7763	4.7369
36	0.0253	−0.1129	3.1812	9.8653	−10.8527	4.7380	4.5969	4.6061
40	−0.1299	−0.3529	3.2500	9.3028	−9.5338	4.4812	4.5039	4.4873
41	0.2345	−0.3887	3.2308	9.8765	−6.4561	4.4515	4.3783	4.4087
42	−0.0532	−0.3780	3.3172	0.0000	−6.8101	4.3166	4.2233	4.2380
43	−0.0593	−0.3637	3.2420	0.0000	−6.0887	4.3548	4.3528	4.3916
44	−0.0509	−0.2910	3.2334	0.0000	−5.8163	4.4938	4.4093	4.4637
45	−0.0173	−0.2675	3.4411	0.0000	−4.9885	4.1204	4.1692	4.1627
46	−0.0032	−0.3884	3.2356	9.3450	−5.2325	4.4109	4.5581	4.5088
2	−0.0370	−0.0890	3.1222	9.5400	−19.7602	4.3608	4.4273	4.4454
3	−0.0755	−0.0701	3.1767	0.0000	−22.6759	4.1360	4.0753	4.0245
Test set								
8	−0.0331	0.0074	3.4042	0.0000	−7.1124	4.3555	4.3170	4.2924
15	−0.1179	−0.1798	3.1493	9.1528	−12.0965	4.4885	4.6353	4.6541
19	−0.0094	−0.2410	3.2785	10.2490	−10.0158	4.5391	4.4604	4.4550
27	0.2318	−0.0409	3.1836	9.3299	−6.6436	4.5577	4.6231	4.6151
30	0.1521	−0.0420	3.1972	9.6832	−5.9395	4.5522	4.6900	4.6686
31	0.1428	−0.0987	3.1981	9.7056	−8.2064	4.6925	4.5884	4.5832
34	0.1890	−0.1345	3.2559	8.9286	−7.2527	4.4983	4.4775	4.4855
37	−0.0381	−0.1129	3.1677	9.6650	−12.0965	4.5832	4.6105	4.6322
38	−0.0316	−0.1254	3.2398	0.0000	−10.6340	4.3739	4.3280	4.3379
39	−0.0351	−0.1352	3.1083	9.3488	−12.6016	4.5969	4.6454	4.6661
47	0.1550	−0.3682	3.2420	10.2298	−8.3332	4.2594	4.3764	4.4001
48	−0.0830	−0.3679	3.2461	9.6983	−6.9305	4.4533	4.5630	4.5202
4	−0.0671	−0.0614	3.1215	0.0000	−19.7602	4.1913	4.2386	4.1875

**Table 7:** Correlation statistics of the model descriptors.

Descriptor	ATSC6c	MATS3i	SpMax5_Bhe	minsOH	VE3_D	VIF	Mean Effect
ATSC6c	1	0.424442	-0.0901	-0.0221	0.3691	2.0195	+0.00265
MATS3i		1	-0.3668	0.0944	-0.3213	1.8603	+0.02267
SpMax5_Bhe			1	-0.2862	0.4360	1.5680	+0.9381
minsOH				1	0.0353	1.1799	-0.0380
VE3_D					1	2.1816	+0.0744

The VIF was computed for each model descriptor, and their scores fall within the threshold limit (VIF< 10) suggesting void multicollinearity which implies that each descriptor is orthogonal to one another (Thompson et al., 2017).

The relative importance of the model descriptors based on their magnitude and direction were computed via the mean effect (ME) approach using Eq. (15).

(15) $$\text{ME}=\frac{\beta_{i}\;\sum_{i}^{n}D_{i}}{\sum_{i}^{n}\left(\beta_{i}\;\sum_{i}^{n}D_{i}\right)}\;$$

Where *βi* represents the coefficient of the descriptor *i* and *Di* represent each descriptor score for a molecule and n represents the number of training set molecules (Wang et al., 2018). It was observed that the SpMax5_Bhe descriptor has the highest positive mean effect score of 0.9381. This suggested that ***SpMax5_Bhe*** has the greatest degree of contribution towards the activity predictions. The predictive potency of the 2D-QSAR models was demonstrated through the graphical scatter plots of experimental versus predicted response activity as shown in Figure 4, and the regression coefficient (R^2^ > 0.6) indicates reliability and the strength of the model proposed.

**Figure 4:** Graphical plot of the experimental against predicted response (pIC_50_).

Model error predictions (residuals) consist of three (3) important components such as random (variance), systematic (bias), and measurement (noise) error, but models are more affected by systematic errors (Shirvani and Fassihi, 2021). Therefore, a model with high systematic error should be reconstructed again to reduce the high level of bias. This is because bias redirects the data into an artificial course that could lead to the wrong interpretation (Umar et al., 2019). The predictive competency of the 2D-QSAR model to predict the reported experimental response activities without any computational errors was determined by exploring the residual plot as shown in Figure 5. Since all the residual values fall within the definite threshold of ±2.5. Hence, it implies that the model is free of systematic error and can give a good prediction.

**Figure 5:** Graphical plot of the standardized residuals versus response (pIC_50_).

### 3.2 Interpretation of the molecular descriptors

**ATSC6c** descriptor is the centered Broto-Moreau autocorrelation-lag 6/weighted by charges which belongs to the spatial autocorrelation parameter in molecular graph theory. It is a 2D-autocorrelation descriptor relating to atomic properties, such as charges, polarizability, electronegativity, and atomic masses (Gonçalves et al., 2020). **MATS3i** is a 2D-autocorrelations descriptor (Moran autocorrelation-lag3/weighted by first ionization potential) that corresponds with the molecular topology, structural features, and atomic properties such as carbon-scaled atomic polarizability, intrinsic state, and van der Waals volume (Altaf et al., 2022). It has a negative coefficient in the model, which implies that the first ionization potential decreases as the inhibitory activity score increases. **SpMax5_Bhe** descriptor is computed by determining the largest absolute eigenvalue of a modified Burden matrix (n = 5) weighted by relative Sanderson electronegativities (Ibrahim et al., 2020). It has the greatest degree of contribution with a positive influence on bioactivity due to its positive mean effect. The descriptor is related to the positive influence of the electronegative features on bioactivity.

The **mins-OH** is the minimum atom-type E-state of –OH groups in a molecular graph. It is a 2D descriptor that represents the electrotopological state for atom type which provides a more accurate and chemically expressive meaning to the role of functional groups, such as –OH, in molecules. Hence, it can be easily described as the addition of –OH groups to the molecular graph increases, the polarity of molecules which makes it more hydrophilic and prevent its cellular membrane uptake (Sanyal et al., 2019). VE3_D is the logarithmic coefficient sum of the last eigenvector from the Barysz matrix (n = 3) weighted by atomic number. The Barysz distance matrix is derived from a vertex and edge-weighted molecular graph that can identify the presence of atoms with more electronegativity (Sanyal et al., 2019).

### 3.3 Model applicability domain of the 2D-QSAR model

The applicability domain of the 2D-QSAR model in chemical space where the model can make a reliable prediction based on the five (5) defined model descriptors stated earlier. In this study, the leverage approach was applied to examine the chemical space. The standardized residuals computed by the GFA-ANN model were plotted against the leverage values for all molecules (Williams plot) to identify the response and structural outliers as presented in Figure 6. Interestingly, all molecules in the dataset were observed to be confined within the standardized residual threshold limit of ±2.5 while, only molecules 4, 8, 47, and 48 were seen to exceed the threshold leverage (h∗) of 0.514. Thus, these influential compounds cannot be considered as templates for designing more prominent molecules with enhanced activities.

**Figure 6:** Scatter plot of the leverage scores against standardized residuals of the GFA-ANN model (Williams plot).

### 3.4 3D-QSAR models validation results

The CoMFA and CoMSIA models were generated for the 48 molecules of 5-benzyl-4-thiazolinone derivatives as anti-influenza inhibitors targeting the H1N1 subtype. The optimized structures were automatically split based on the structural diversity method into model building set (35 as training set) and test set (13 validation set) using Sybyl-X 2.1.1. The validation parameters for all possible CoMFA models were shown in Table 8. Among the possible CoMFA models generated, the CoMFA_ES model with acceptable statistical validation metrics as Q^2^ (0.5390), ${\text{R}}_{\text{train ​}}^{2}$ (0.9039), SEE (0.0615), and ${\text{R}}_{\text{test}}^{2}$ (0.5386) was selected as the best model.

**Table 8:** Statistical validation results of probable CoMFA models.

Descriptors	Q^2^	R^2^	SEE	N
Steric (S)	0.412	0.837	0.0773	3
Electrostatic (E)	0.409	0.918	0.0575	3
S + E	0.539	0.903	0.0615	5

Q^2^: Leave one out cross-validated correlation coefficient.

R^2^: Non-cross validated correlation coefficient.

SEE: Standard error of estimation.

N: number of optimum components.

Similarly, 30 possible CoMSIA models based on the five (5) different field descriptors combination which include, steric (S), electrostatics (E), hydrophobic (H), and hydrogen bond donor (D), and hydrogen bond acceptors (A) were shown in Table 9. Furthermore, four (4) CoMSIA models were identified as the best models out of the possible models generated because of their acceptable validation parameters. However, the CoMSIA_EA model was selected as the best model with the computed validation metrics (Q^2^ = 0.547 with 4 components, the R^2^ value of 0.888, and a relatively low SEE value of 0.0673). In addition, the validations metrics of the best CoMFA and CoMSIA models (Table 10) were found within the benchmark scores for an acceptable QSAR model that was proposed by Alexander Golbraikh and Alexander Tropsha (Q^2^ > 0.5 and R^2^ > 0.6). This implies that the validation metrics of the models generated are statistically reliable which indicates their predictive potential and robustness (Shirvani and Fassihi, 2021).

**Table 9:** Statistical validation results of all possible CoMSIA models.

S/N	Descriptors	Q^2^	R^2^	SEE	N
1	Steric (S)	0.501	0.890	0.0655	5
2	Electrostatic (E)	0.489	0.743	0.0955	2
3	Hydrophobic (H)	0.488	0.707	0.1019	2
4	H-Bond Donor(D)	0.439	0.918	0.0568	5
5	H-Bond Acceptor(A)	0.511	0.875	0.0687	4
6	S + E	0.466	0.714	0.1007	2
7	S + H	0.441	0.823	0.0804	3
8	S + D	0.429	0.940	0.0502	7
9	S + A	0.485	0.883	0.0664	4
10	E + H	0.436	0.734	0.0971	2
11	E + D	0.420	0.843	0.0758	3
12	E + A	0.547	0.880	0.0673	4
13	H + D	0.444	0.943	0.0488	7
14	H + A	0.467	0.856	0.0725	3
15	S + E + H	0.438	0.715	0.1005	2
16	S + E + D	0.419	0.946	0.0477	7
17	S + E + A	0.512	0.874	0.0691	4
18	S + H + A	0.454	0.854	0.0732	3
19	S + H + D	0.364	0.745	0.0951	2
20	S + A + D	0.486	0.952	0.0449	7
21	E + A + D	0.526	0.936	0.0502	5
22	E + A + H	0.498	0.847	0.074	3
23	A + H + D	0.491	0.924	0.054	7
24	E + D + H	0.397	0.828	0.079	3
25	S + E + H + D	0.369	0.775	0.0893	2
26	S + E + H + A	0.480	0.871	0.069	4
27	S + H + D + A	0.475	0.925	0.0542	5
28	E + H + D + A	0.534	0.963	0.0395	7
29	S + E + D + A	0.482	0.941	0.0490	6
30	S + E + H + D + A	0.489	0.959	0.0412	7

**Table 10:** Statistical validation results of the best 3D-QSAR models.

3D-QSAR Models	Q^2^	R^2^	SEE	N	R^2^_test_
CoMFA_E + S	0.539	0.903	0.0615	5	0.5386
CoMSIA_E + A	0.547	0.880	0.0673	4	0.6015
CoMSIA_S + E + A	0.512	0.874	0.0691	4	0.6276
CoMSIA_E + A + D	0.526	0.936	0.0502	5	0.6041
CoMSIA_E + H + D + A	0.534	0.963	0.0395	7	0.6890

The scatter plots of experimental against predicted inhibitory activities (pIC_50_) for the training and test set molecules of both CoMFA and CoMSIA models revealed a good linear correlation, as presented in Figures 7a and 7b respectively. Also, the systematic error predictions in the models were assessed using the standardized residual versus experimental inhibitory activity plots as shown in Figs 8a-b. Hence, the standardized residual plots for both 3D-QSAR models revealed a random scattering above and below the zero baselines which is an indication of the non-existence of systematic (bias) error in the studies.

**Figure 7:** Scatter plot of the predicted pIC_50_ against experimental pIC_50_ (a) CoMFA model, (b) CoMSIA model.

**Figure 8:** Scatter plot of the standardized residuals against experimental pIC_50_ (a) CoMFA_ES model (b) CoMSIA_EA model.

#### 3.4.1 Contour map analysis of the CoMFA and CoMSIA models

The contour map interpretation of the CoMFA and CoMSIA models generated is one of the most attractive aspects of the 3D-QSAR analysis which involves the visualization of all favoured and disfavoured regions of the molecular fields surrounding the molecules as bioactivities functions (ElMchichi et al., 2020). **Molecule 11** with the highest activity was chosen as a template to examine the most prominent field contributions for the studied dataset. The CoMFA steric and electrostatic contour maps of **molecule 11** were shown in Figs. 9A-B. The green contours signified that the desirable addition of bulky groups in the regions would increase the activity, while the yellow contours depicted that bulky groups are undesirable in the region for increasing activity (Gu et al., 2021). Green contours are predominantly distributed on the ethyl acetate and 2-methoxy substituents of **molecule 11**, proposing that the introduction of bulkier groups in these regions would have enhanced the activity. Meanwhile, the yellow contours were distributed around the oxygen of the same methoxy substituent of the molecule, indicating that further attachment of bulkier fragments to the group's region would cause a decrease in the activity of the molecule. The electrostatic contour maps for the CoMFA model revealed the red contour regions where negatively charged groups are desirable and the blue contour areas are positively charged favoured regions for increasing activity. The red contour maps were observed near the ends of the substituents such as oxygens of ethyl acetate, methyl group attached to the thiazole moiety, hydroxyl (4-OH) and methoxy (3-OCH_3_) groups of the benzene moiety of **molecule 11**, while the central surface of the molecule was enclosed with blue contours. The blue contour fields indicate that the further addition of positively charged substituents could lead to an increase in the activity of the molecule.

**Figure 9:** 3D fields of the CoMFA_ES model for the most active compound (molecule 11), (A) green areas depict desirable steric bulk while yellow areas disfavours steric bulk, (B) electrostatic contour map where blue regions favours positive charge and red regions favours negative charge.

Furthermore, the red contours around the molecular ends suggest that more electronegative substituents should be attached to the regions for enhanced activity. However, these predictions were consistent with the electrostatic contour map for the CoMSIA_EA model generated. The contour maps for the CoMSIA_EA model with electrostatic and hydrogen bond acceptor field contributions were shown in Figs. 10A-B. From the HBA contours map, the magenta contours reveal the favorable HBA regions while the red contours show the unfavorable HBA regions. As such, the red contour was observed near the oxygen (-O-) of the ethyl acetate substituent attached to thiazole moiety while the magenta contours were observed near carbonyl oxygen (C=O) of the ethyl acetate, and the hydroxyl oxygen (4-OH) of benzene moiety of the same molecule.

**Figure 10:** 3D fields contribution of the CoMSIA_EA model for the most active compound (molecule 11), (A) magenta contours represent regions for desirable hydrogen bond acceptors while red areas represent undesirable acceptors, (B) electrostatic contour map where blue regions favours positive charge and red regions favours negative charge.

The general depiction of the contour maps from the CoMFA and CoMSIA models were summarized in Figure 11. The outcome of these analysis reaffirmed the largest influence of the 4-position substituents of thiazole on the activities as reported by Xiao et al. (2021). However, the addition of more substituted benzyl methylene with more electronegative and steric groups to the 5-position of the 4-thiazolinone ring may enhance the inhibitory activity of the molecules.

**Figure 11:** Summary of the 3D-QSAR analysis.

### 3.5 Molecular docking studies

Molecular docking simulation is an important molecular modelling strategy in the computer-assisted design of new molecules (structure-based drug design) which evaluates the binding interactions between the small molecules (ligands) and the targeted protein (Ibrahim et al., 2020). The 48 molecules of the dataset were docked into the active pocket of pH1N1 neuraminidase (PDB: 3TI5) using MOE software. The co-crystalized zanamivir of the protein was extracted and re-docked into the binding pocket to confirm the reliability of the docking algorithm used by the MOE program as well as to note the amino acid residues surrounding the ligand. The binding affinities of the molecules and zanamivir were summarized in Table 11. The results revealed the docking energies of the best poses ranging from −8.2964 to −6.4392 kcal/mol which confirms their robust potency in comparison with zanamivir, indicating that most of the studied molecules have higher binding capacity than zanamivir. However, six (6) leads (9, 10, 11, 17, 22, and 31) with relatively high activity (pIC_50_ ≥ 4.50) and docking score (≥−7.5 kcal/mol) were identified as the possible lead candidates for future exploration of improved anti-influenza agents. **Molecule 11** as the most potent molecule with the highest pIC_50_ of 4.8841 revealed a good docking score of −7.5022 kcal/mol, and the residual profile the complex formed was visualized in Figure 12.

**Table 11:** Molecular docking energies of 5-benzyl-4-thiazolinone derivatives (1–48) and zanamivir with pH1N1 neuraminidase receptor.

S/N	Score	rmsd_refine	E_conf	E_place	E_score1	E_refine	E_score2
1	-6.9831	1.8152	-73.7490	-69.6008	-10.1108	-39.4165	-6.9831
2	-6.9824	5.1927	-218.3650	-76.6869	-14.4964	-41.1106	-6.9824
3	-6.8311	1.3184	-247.8260	-86.0685	-14.6259	-38.8715	-6.8311
4	-6.7030	1.2569	-242.0660	-86.1565	-14.4032	-37.7068	-6.7030
5	-7.1048	1.4906	-219.2830	-77.6698	-14.2432	-42.7637	-7.1048
6	-6.9620	2.1954	-209.3300	-81.9871	-14.8346	-34.3155	-6.9620
7	-7.2487	2.1961	-213.7020	-68.4690	-13.9033	-41.1331	-7.2487
8	-7.5203	0.8862	-236.4350	-96.0306	-14.7716	-40.9864	-7.5202
9	-7.6306	1.8323	-202.1330	-62.6307	-14.0400	-43.4870	-7.6306
10	-7.8816	1.9186	-283.3290	-70.9370	-13.8800	-47.0044	-7.8816
11	-7.5022	1.4998	-224.3970	-84.6704	-14.9998	-38.2096	-7.5022
12	-7.1972	1.7001	-247.1960	-82.3165	-16.3960	-42.5298	-7.1972
13	-7.3260	1.2654	-240.2570	-62.7389	-15.6182	-45.2596	-7.3260
14	-6.4393	3.3371	-838.6300	-93.1821	-20.9030	-25.2268	-6.4393
15	-6.6507	1.3029	-254.1110	-71.0366	-14.7685	-38.2769	-6.6507
16	-7.0622	1.1356	-209.8560	-84.3116	-14.3066	-43.9421	-7.0622
17	-7.5775	1.8048	-256.3010	-79.4413	-16.7853	-46.0432	-7.5775
18	-7.0222	1.4287	-227.0220	-56.5362	-14.4892	-43.4416	-7.0222
19	-7.5512	1.1467	-189.0950	-73.7108	-15.2324	-41.3378	-7.5512
20	-7.1072	1.6515	-210.3830	-72.2574	-16.1456	-40.3821	-7.1072
21	-7.3026	1.7640	-205.6890	-50.3991	-16.1187	-46.0320	-7.3026
22	-7.8240	1.6129	-192.2170	-94.2830	-15.1027	-47.1838	-7.8240
23	-7.4310	1.8469	-203.3440	-49.0440	-17.0886	-46.2254	-7.4310
24	-7.0948	2.0346	-549.3960	-42.1918	-16.4244	-39.3711	-7.0948
25	-6.8982	1.7889	-257.5520	-79.3323	-13.5534	-35.5172	-6.8982
26	-7.5742	1.8526	-88.8226	-93.2651	-11.9930	-44.3407	-7.5742
27	-6.7739	3.7520	-92.6378	-69.6697	-11.1069	-39.7212	-6.7739
28	-7.5149	2.3913	-66.1309	-55.8518	-11.1113	-44.0013	-7.5149
29	-7.6113	1.5941	-80.2895	-87.8352	-11.1546	-44.9662	-7.6113
30	-7.4709	1.5039	-80.2671	-96.5625	-11.2925	-45.3060	-7.4709
31	-7.9066	1.9585	-79.2294	-67.6142	-11.9116	-45.4157	-7.9066
32	-7.0262	1.5950	-56.6493	-73.3923	-10.6632	-38.7261	-7.0262
33	-6.4774	1.3395	-100.6380	-65.3704	-10.9371	-37.8411	-6.4773
34	-6.7005	2.3201	-96.0212	-86.1006	-11.0682	-40.4141	-6.7005
35	-6.3790	2.2068	-99.7614	-95.6545	-10.6303	-36.2379	-6.3790
36	-6.7085	2.4881	-79.3080	-83.8075	-11.1555	-38.5037	-6.7085
37	-6.6722	1.3170	-86.4799	-88.0450	-10.9725	-40.0835	-6.6722
38	-6.6224	1.0649	-74.7140	-91.0756	-10.9740	-40.2328	-6.6224
39	-6.6070	2.2338	-67.8629	-71.5647	-12.5070	-30.0313	-6.6070
40	-6.5010	2.1024	-70.2952	-93.2770	-11.8520	-37.0667	-6.5010
41	-7.1805	1.1736	-59.6742	-68.3012	-11.3095	-41.5516	-7.1805
42	-7.5998	1.2680	-32.5972	-98.3048	-11.6669	-43.5905	-7.5998
43	-7.6408	1.3351	-62.0518	-93.3567	-11.3797	-44.5894	-7.6408
44	-7.1438	1.5098	-57.2174	-87.1503	-10.8695	-41.1641	-7.1438
45	-8.2964	1.4888	-112.8360	-100.8420	-11.9067	-51.6596	-8.2964
46	-7.2227	1.6196	-72.0725	-66.8217	-11.5112	-41.7903	-7.2227
47	-7.0413	1.8996	-46.7257	-63.9331	-11.2684	-36.3190	-7.0413
48	-7.8066	1.7015	-61.8125	-90.4101	-12.4004	-45.4162	-7.8065
Zanamivir	-7.4222	1.572874	-354.562	-91.0359	-20.3477	-57.1482	-7.42222

Score: the final docking score, rmsd_refine: the root means square deviation between the pose before and after refinement, E_conf: the energy of the conformer. E_refine: core from the refinement stage, calculated to be the sum of the van der Waals electrostatics and solvation energies, under the Generalized Born solvation model (GB/VI), E_score1: Score from rescoring stages 1, E_place: Score from the placement stage, E_score2: Score from rescoring stages 2.

**Figure 12:** 3D docking view of molecule 11 with the pH1N1 neuraminidase protein (PDB: 3TI5): (A) the best binding mode of molecule 11, (B) 3D hydrogen bond surfaces around the molecule (C) 2D residual interaction of 11-complex, (D) 2D residual interaction of zanamivir complex.

The active site of the pH1N1 neuraminidase (PDB:3TI5) protein contains 19 conserved residues of amino acids where eight among them (ARG118, ARG152, ARG224, ARG292, ARG371, ASP151, GLU276, and TYR406) are highly conserved and can directly interact with the substrate. The remaining 11 amino acid residues (GLU119, ARG156, TRP178, SER179, ASN294, ILE222, GLU227, THR225, GLU277, LEU134, and SER246) behave as scaffolds for the stabilization of the active site conformation. The best binding modes of **molecule 11** in the binding site (11-complex) revealed four (4) conventional H-bonds, three (3) carbon-H bonds, seven (7) electrostatic, four (4) hydrophobic, and two (2) other interaction types with different active amino acid residues as summarized in Table 12. The analysis of the residual interactions revealed 4 complicated networks of hydrogen bond interactions with the amino acid residues of A: ARG118, A: ARG371, A: ARG371, and A: GLU227 at different bond distances of 3.0003 Å, 2.7684 Å, 2.3066 Å, and 1.8321 Å respectively. The molecule formed 5 different electrostatic interactions due to strong attractive positive charges from the active residues such as A: ARG118, A: ARG292, and A: ARG371, while π-cation and π-anion interactions were conversely formed with A: ARG371 and A: GLU277 respectively. For the hydrophobic interaction, the 2-EtO group of the molecule interacts with the alkyl group of ILE149 to form one (1) alkyl-alkyl hydrophobic interaction type at a distance of 4.3738 Å, while the remaining 2-hydrophobic interactions formed were as a result of the π-alkyl interaction type with ARG225 and PRO431 residues at 5.4696 Å and 4.4297 Å interaction distances respectively. The residual interactions between the thiazole moiety of **molecule 11** and highly conserved amino acids in this study are weaker than that of zanamivir as observed in other related studies (Lu and Chong, 2012; Meng et al., 2016; Selvaraj et al., 2020; Wang et al., 2017; Xiao et al., 2021). Also, this is in agreement with our 3D-QSAR studies suggesting that the thiazole moiety may not have a significant effect on NA inhibitory activity. The conventional hydrogen bond interactions with ARG118, GLU227, and ARG371 significantly made 5-benzylidenethiazolinone moiety more stable in both SA-cavity and 430-loop cavity accordingly. This tenders an important route for the exploration of more highly potent NA inhibitors targeting both 150 and 430-loop cavities respectively.

**Table 12:** Binding interactions of molecule 11 with the active site of pH1N1 neuraminidase.

Bond Distance (Å)	Interaction type	From	Chemistry	To	Chemistry
4.95601	Electrostatic	A: ARG118	Positive	11	Negative
5.01423	Electrostatic	A: ARG118	Positive	11	Negative
4.61425	Electrostatic	A: ARG292	Positive	11	Negative
5.19025	Electrostatic	A: ARG292	Positive	11	Negative
3.54855	Electrostatic	A: ARG371	Positive	11	Negative
3.00036	Hydrogen Bond	A: ARG118	H-Donor	11	H-Acceptor
2.76845	Hydrogen Bond	A: ARG371	H-Donor	11	H-Acceptor
2.30669	Hydrogen Bond	A: ARG371	H-Donor	11	H-Acceptor
1.83219	Hydrogen Bond	11	H-Donor	A: GLU227	H-Acceptor
2.68284	Carbon H-Bond	A: ARG371	H-Donor	11	H-Acceptor
2.98371	Carbon H-Bond	11	H-Donor	A: GLU276	H-Acceptor
3.29475	Other (Sulfur-X)	11	Sulfur	A: TYR406	O, N, S
3.12597	Electrostatic	A: ARG371	Positive	11	Pi-Orbitals
3.46195	Electrostatic	A: GLU277	Negative	11	Pi-Orbitals
3.4012	C–H bond (Pi-Donor)	A: TYR406	H-Donor	11	Pi-Orbitals
5.16441	Other (Pi-Sulfur)	11	Sulfur	A: TYR406	Pi-Orbitals
3.7482	Hydrophobic (Alkyl)	11	Alkyl	A: ARG371	Alkyl
4.05516	Hydrophobic (Alkyl)	11	Alkyl	A: LYS432	Alkyl
5.20931	Hydrophobic (Pi-Alkyl)	A: TRP403	Pi-Orbitals	11	Alkyl
5.1745	Hydrophobic (Pi-Alkyl)	11	Pi-Orbitals	A: PRO431	Alkyl

### 3.6 Drug likeness assessment and ADMET prediction

In assessing the drug-likeness of the molecules, the physicochemical parameters of the molecules are usually related to some filter variants. Therefore, relevant physicochemical parameters (Figure 13) generated from the ADMETlab 2.0 web server were assessed using numerous drug-likeness rules such as Lipinski’s rule, Pfizer’s rule, GSK’s rule, and Golden triangle rule as presented in Table 13.

**Figure 13:** Physicochemical radar chart of the selected lead compounds in the dataset.

**Table 13:** Drug likeness parameters of 5-benzyl-4-thiazolinone derivatives appraised by Lipinski, Pfizer, GSK, and Golden Triangle rules.

S/N	MW	Dense	LogS	LogD	LogP	nHA	nHD	nRot	TPSA	Lipinski	Pfizer	GSK	Golden Triangle
1	389.05	1.086	-4.361	2.891	2.747	7	2	5	104.11	Accepted	Accepted	Accepted	Accepted
2	389.05	1.086	-3.832	2.294	2.513	7	2	5	104.11	Accepted	Accepted	Accepted	Accepted
3	403.07	1.073	-4.763	2.766	2.919	7	1	6	93.11	Accepted	Accepted	Rejected	Accepted
4	391.05	1.1	-4.683	2.616	2.966	6	1	5	83.88	Accepted	Accepted	Accepted	Accepted
5	407.02	1.116	-4.84	3.169	3.46	6	1	5	83.88	Accepted	Accepted	Rejected	Accepted
6	417.05	1.092	-3.91	1.928	2.762	8	2	6	121.18	Accepted	Accepted	Rejected	Accepted
7	431.06	1.08	-4.877	2.483	2.99	8	1	7	110.18	Accepted	Accepted	Rejected	Accepted
8	430.08	1.072	-4.723	2.392	2.329	8	2	7	112.98	Accepted	Accepted	Rejected	Accepted
9	389.05	1.086	-4.003	2.675	2.461	7	2	5	104.11	Accepted	Accepted	Accepted	Accepted
10	419.06	1.09	-4.697	2.671	2.588	8	2	6	113.34	Accepted	Accepted	Rejected	Accepted
11	419.06	1.09	-4.455	2.605	2.401	8	2	6	113.34	Accepted	Accepted	Rejected	Accepted
12	405.05	1.103	-3.659	2.663	2.487	8	3	5	124.34	Accepted	Accepted	Rejected	Accepted
13	405.05	1.103	-3.716	2.378	2.187	8	3	5	124.34	Accepted	Accepted	Rejected	Accepted
14	479.02	1.168	-4.292	2.208	2.73	13	2	7	190.39	Accepted	Accepted	Rejected	Accepted
15	391.03	1.118	-2.965	1.474	1.778	8	3	4	124.34	Accepted	Accepted	Accepted	Accepted
16	405.05	1.103	-4.305	2.342	2.025	8	2	5	113.34	Accepted	Accepted	Rejected	Accepted
17	447.09	1.067	-4.842	2.81	3.071	8	2	6	113.34	Accepted	Accepted	Rejected	Accepted
18	403.07	1.073	-4.375	2.943	2.788	7	2	5	104.11	Accepted	Accepted	Rejected	Accepted
19	433.08	1.078	-4.976	2.926	2.949	8	2	6	113.34	Accepted	Accepted	Rejected	Accepted
20	419.06	1.09	-4.033	2.565	2.483	8	3	5	124.34	Accepted	Accepted	Rejected	Accepted
21	433.08	1.078	-4.725	2.854	2.704	8	2	6	113.34	Accepted	Accepted	Rejected	Accepted
22	463.09	1.082	-5.097	2.663	2.604	9	2	7	122.57	Accepted	Accepted	Rejected	Accepted
23	447.09	1.067	-4.771	3.128	3.211	8	2	8	113.34	Accepted	Accepted	Rejected	Accepted
24	418.04	1.113	-4.531	2.731	2.512	9	1	7	127.02	Accepted	Accepted	Rejected	Accepted
25	388.07	1.076	-3.81	1.918	2.093	7	3	6	109.9	Accepted	Accepted	Accepted	Accepted
26	417.05	1.092	-3.795	1.806	2.516	8	2	7	121.18	Accepted	Accepted	Rejected	Accepted
27	389.05	1.086	-3.592	2.595	2.271	7	2	6	104.11	Accepted	Accepted	Accepted	Accepted
28	419.06	1.09	-4.484	2.585	2.383	8	2	7	113.34	Accepted	Accepted	Rejected	Accepted
29	419.06	1.09	-4.012	2.195	2.256	8	2	7	113.34	Accepted	Accepted	Rejected	Accepted
30	419.06	1.09	-4.137	2.506	2.212	8	2	7	113.34	Accepted	Accepted	Rejected	Accepted
31	433.08	1.078	-4.584	2.771	2.571	8	2	7	113.34	Accepted	Accepted	Rejected	Accepted
32	388.03	1.11	-4.007	2.433	2.243	8	1	4	117.79	Accepted	Accepted	Accepted	Accepted
33	359.04	1.081	-3.33	2.047	2.062	6	2	3	94.88	Accepted	Accepted	Accepted	Accepted
34	387.03	1.088	-3.481	1.56	2.216	7	2	4	111.95	Accepted	Accepted	Accepted	Accepted
35	359.04	1.081	-3.392	2.449	2.006	6	2	3	94.88	Accepted	Accepted	Accepted	Accepted
36	389.05	1.086	-3.76	2.045	1.998	7	2	4	104.11	Accepted	Accepted	Accepted	Accepted
37	389.05	1.086	-3.784	2.398	1.955	7	2	4	104.11	Accepted	Accepted	Accepted	Accepted
38	387.03	1.106	-4.237	2.333	2.175	7	1	3	93.11	Accepted	Accepted	Accepted	Accepted
39	375.03	1.1	-3.086	2.06	1.734	7	3	3	115.11	Accepted	Accepted	Accepted	Accepted
40	432.06	1.1	-3.909	2.786	3.669	9	2	5	138.02	Accepted	Accepted	Rejected	Accepted
41	404.06	1.094	-4.711	3.609	3.847	8	2	4	120.95	Accepted	Accepted	Rejected	Accepted
42	433.05	1.12	-4.891	3.672	3.86	10	1	5	143.86	Accepted	Accepted	Rejected	Accepted
43	418.08	1.081	-5.273	3.81	4.005	8	1	5	109.95	Accepted	Accepted	Rejected	Accepted
44	406.06	1.108	-5.162	3.797	4.06	7	1	4	100.72	Accepted	Accepted	Rejected	Accepted
45	445.09	1.08	-5.124	2.798	3.423	9	2	6	129.82	Accepted	Accepted	Rejected	Accepted
46	404.06	1.094	-4.388	3.377	3.501	8	2	4	120.95	Accepted	Accepted	Rejected	Accepted
47	434.07	1.098	-4.905	3.297	3.687	9	2	5	130.18	Accepted	Accepted	Rejected	Accepted
48	434.07	1.098	-4.738	3.231	3.431	9	2	5	130.18	Accepted	Accepted	Rejected	Accepted

Key: MW: Molecular Weight, Log P: Logarithm of the n-octanol/water distribution coefficient, Log S: Logarithm of aqueous solubility value, Log D: Logarithm of the n-octanol/water distribution coefficient at pH = 7.4, nHA: Number of hydrogen bond acceptors, nHD: Number of hydrogen bond donors, TPSA: Topological polar surface area, nRot: Number of rotatable bonds, nRing: Number of rings, MaxRing: Number of atoms in bigger rings, nHet: Number of heteroatoms, fChar: Formal charge, nRig: Number of rigid bond.

The physicochemical properties for the six lead compounds (9, 10, 11, 17, 22, 31) are within the upper limit (brown) and lower limit (red) as presented in the radar charts accordingly (Figure 13). The six lead molecules which have passed the Lipinski rule of five **(**Table 14**)** were further assessed with other drug-likeness filter rules such as the Ghose filter rule, Veber’s rule, Egan’s rule, and Muegge’s rule using the SwissADME web server as shown in Table 15. Lipinski's criteria for drug-likeness include molecular weight (MW ≤ 500 g/mol), n-octanol/water distribution coefficient (Log P ≤ 5), number of hydrogen bond acceptors (nHA ≤10), and number of hydrogen bond donors (nHD ≤5) (Ahmed et al., 2022; Chauhan et al., 2014). From Lipinski's table of the lead molecules in the data set, the Log P scores of the molecules are relatively close to 3 log mol/L (optimal limit) except for **molecule 17** which is slightly above the optimal limit (0 < Log P < 3). This implies that the molecules have low aqueous solubility and good oral bioavailability (Adianingsih et al., 2022; Arámburo-Gálvez et al., 2022). The Log P also gives information on the cellular membrane permeability and hydrophobic binding to macromolecules such as the target receptors, plasma proteins, metabolizing enzymes, or transporters (Dowdy et al., 2022). Zanamivir and oseltamivir standard neuraminidase drugs have lower Log P scores of 1.013 and -1.317 which tend to experience difficulty in penetrating the lipid bilayer of the cell membrane.

**Table 14:** Lipinski’s rule of the lead molecules in the dataset.

Molecule	MW (g/mol)	Log P (log mol/L)	nHA	nHD	nLV
9	389.05	2.461	7	2	0
10	419.06	2.588	8	2	0
11	419.06	2.401	8	2	0
17	447.09	3.071	8	2	0
22	433.08	2.604	8	2	0
31	433.08	2.571	8	2	0
Oseltamivir	330.15	-1.317	10	9	0
Zanamivir	312.2	1.013	6	3	0
Rule	≤500	≤5	≤10	≤5	≤1

Key: Molecular weight (MW), n-octanol/water distribution coefficient (Log P), number of hydrogens bond acceptors (nHA), number of hydrogen bond donors (nHD), Number of Lipinski violations (nLV).

**Table 15:** Drug likeness assessment of the lead compounds based on Ghose, Veber, Egan, Muegge, QED, and Synthetic accessibility scores.

Molecule	Ghose	Veber	Egan	Muegge	QED	SA score
9	Yes	No	No	No	0.62	3.148
10	Yes	No	No	No	0.582	3.215
11	Yes	No	No	No	0.582	3.158
17	Yes	No	No	No	0.549	3.25
22	Yes	No	No	No	0.515	3.32
31	Yes	No	No	No	0.554	3.272
Oseltamivir	Yes	Yes	Yes	Yes	0.213	4.392
Zanamivir	Yes	Yes	Yes	Yes	0.691	3.758

Key: Quantitative Estimate of Drug-likeness (QED), Synthetic accessibility (SA) score.

The lead molecules were also appraised for their quantitative estimate of drug-likeness (QED), synthetic accessibility scores, and other drug-likeness rules such as Ghose, Veber, Egan, and Muegge rules. The QED scores of the lead molecules are less than 0.67 signifying unattractive measures as drug-like compounds (Bickerton et al., 2012), but they are predicted to be easily synthesized due to their low SA scores of less than 6. The lead molecules were able to satisfy the Ghose rule only among the other drug-likeness rules as shown in Table 15.

The biochemical processes involved from the administration of a drug into the body to its elimination play an important role in lead identification and optimization (Hossen et al., 2022). A perfect drug candidate must be non-toxic, and when administered should be absorbed into the circulatory system and eradicated without affecting the biological activity (Hossen et al., 2022). These discrete biochemical processes are closely interrelated leading to the evaluation of ADMET properties as one of the prime factors in the process of drug discovery (Xu, 2022). The six lead molecules were further subjected to the ADMET prediction using the ADMETlab 2.0 web server as mentioned earlier. Some of the relevant computed ADMET parameters include human intestinal absorption (HIA), human colon adenocarcinoma cell lines (Caco-2) permeability, Madin−Darby Canine Kidney cells (MDCK) permeability, plasma glycoprotein (Pgp) inhibitor, plasma glycoprotein (Pgp) substrate, plasma protein binding (PPB), volume distribution (VD), blood-brain barrier (BBB) penetration, human cytochromes (CYP), clearance (CL), half-life (T1/2), AMES toxicity, carcinogenicity (Carc), eye irritation (EI), respiratory toxicity (RT) as shown in Table 16. The Caco-2 cell permeability has been an important index for an eligible drug candidate which is associated with human intestinal absorption (Ahmed et al., 2022). The lead compounds were considered to have proper Caco-2 cell permeability because their values are higher than the optimal score of 5.15 log cm/s. The computed values for HIA showed that **molecules 9 and 10** have excellent probability of absorption in the intestinal membrane. **Molecules 11 and 31** were predicted to have moderate absorption, while **molecules 17 and 22** tend to be poorly absorbed (>0.7). The MDCK permeability is utilized as an in-vitro model for permeability screening, and its apparent coefficient is used to assess the efficiency of chemicals in the body, and also to estimate the effect of the blood-brain barrier. The lead compounds were considered to have high passive MDCK permeability with predicted coefficients of greater than 2.0 × 10^−5^ cm/s. The output results of the lead molecules revealed an excellent probability of being Pgp non-inhibitor and Pgp non-substrate whose range of values are within 0 and 1. PPB is one of the most important mechanisms of drug uptake and distribution resulting from the drug-protein bindings in the plasma which strongly affects the pharmacodynamics behavior of the drug (Xiong et al., 2021). The lead compounds were also predicted to have a high value of PPB (>90%) depicting a broad therapeutic index. The theoretical concept of the VD parameter is used to relate the administered drug dose with the actual initial concentration in the circulatory system which often describes the in-vivo distribution (Xiong et al., 2021). As such, the lead molecules are predicted to have proper VD values in the range of 0.04–20 L/kg. The BBB permeate output of the lead molecules was classified as BBB + category whose predicted values are > -1. For the metabolism, the predicted outputs revealed the probabilities of being either lead substrates or inhibitors of CYPs of the isoenzymes (1A2, 3A4, 2C9, 2C19, and 2D6) whose range of values is within 0–1. The clearance of a drug (CL) is an important pharmacokinetic measure that describes how the drug is excreted from the body. The predicted clearance penetration results of the lead molecules showed that only **molecules 17 and 31** with the probability values of 6.945 and 6.521 mg/min/kg respectively, tend to have moderate clearance (<5 mg/min/kg), while other **molecules (9, 10, 11 and 22)** are predicted to have low clearance levels. In terms of toxicity, the AMES mutagenicity, eye irritation, and respiratory toxicity of the lead compounds were all predicted as non-toxic which is in agreement with the previous reports by Xiao et al. (2021).

**Table 16:** ADMET properties of the lead molecules in the dataset.

Category	Properties	Prediction probability values (symbols)					
		9	10	11	17	22	31
Absorption	HIA	0.034 (---)	0.203 (--)	0.486 (−)	0.813 (++)	0.891 (++)	0.494 (−)
	Caco-2	-4.973	-5.039	-5.045	-4.992	-5.07	-4.921
	MDCK Permeability	1.76 × 10^−;5^	1.75 × 10^−;5^	1.67 × 10^−;5^	1.7 × 10^−;5s^	1.52 × 10^−;5^	1.68 × 10^−;5^
	Pgp-inhibitor	0.001 (---)	0.01 (---)	0.005 (---)	0.136 (--)	0.383 (−)	0.004 (---)
	Pgp-substrate	0 (---)	0 (---)	0.001 (---)	0 (---)	0.001 (---)	0.002 (---)
	PPB	99.19%	100.12%	99.67%	100.72%	99.88%	97.79%
Distribution	VD	0.332	0.416	0.306	0.488	0.28	0.348
	BBB	0.092 (---)	0.027 (---)	0.028 (---)	0.046 (---)	0.017 (---)	0.099 (---)
	CYP1A2 inhibitor	0.908 (+++)	0.874 (++)	0.864 (++)	0.73 (++)	0.648 (+)	0.898 (++)
	CYP1A2 substrate	0.137 (--)	0.864 (++)	0.867 (++)	0.857 (++)	0.973 (+++)	0.776 (++)
	CYP2C19 inhibitor	0.926 (+++)	0.946 (+++)	0.923 (+++)	0.911 (+++)	0.9 (++)	0.956 (+++)
	CYP2C19 substrate	0.065 (---)	0.188 (--)	0.086 (---)	0.128 (--)	0.407 (−)	0.112 (--)
Metabolism	CYP2C9 inhibitor	0.94 (+++)	0.956 (+++)	0.942 (+++)	0.955 (+++)	0.947 (+++)	0.952 (+++)
	CYP2C9 substrate	0.634 (+)	0.791 (++)	0.677 (+)	0.672 (+)	0.581 (+)	0.789 (++)
	CYP2D6 inhibitor	0.287 (--)	0.448 (−)	0.258 (--)	0.413 (−)	0.082 (---)	0.188 (--)
	CYP2D6 substrate	0.164 (--)	0.301 (−)	0.232 (--)	0.19 (--)	0.221 (--)	0.203 (--)
	CYP3A4 Inhibitor	0.413 (−)	0.744 (++)	0.67 (+)	0.642 (+)	0.684 (+)	0.715 (++)
	CYP3A4 substrate	0.265 (--)	0.459 (−)	0.411 (−)	0.383 (−)	0.575 (+)	0.673 (+)
Excretion	CL	4.298	3.835	4.95	6.945	3.83	6.521
	T1/2	0.405	0.307	0.455	0.468	0.588	0.675
	AMES	0.169 (--)	0.288 (--)	0.176 (--)	0.086 (---)	0.021 (---)	0.148 (--)
Toxicity	Carc	0.91 (+++)	0.915 (+++)	0.912 (+++)	0.936 (+++)	0.907 (+++)	0.885 (++)
	EI	0.116 (--)	0.051 (---)	0.058 (--)	0.028 (---)	0.014 (---)	0.022 (---)
	RT	0.245 (--)	0.248 (--)	0.228 (--)	0.395 (−)	0.787 (++)	0.351 (−)

Key: The prediction probability values are classified into six symbols: 0–0.1(---), 0.1–0.3(--), 0.3–0.5(−), 0.5–0.7(+), 0.7–0.9(++), and 0.9–1.0(+++). Generally, ‘+++’ or ‘++’ represents the molecule is more likely to be toxic or defective, while ‘−;−;’or‘−;’ represents nontoxic or appropriate.

## 4 Conclusion

In conclusion, the study utilized some in-silico modelling concepts on 48 analogs of 4-thiazolinone as influenza neuraminidase inhibitors. The 2D-QSAR models (GFA-MLR and GFA-ANN) models with the feature-selected descriptors as MATS3i, SpMax5_Bhe, minsOH, and VE3_D were adopted for predicting NA inhibitory activity (pIC_50_) of the molecules. Similarly, the accepted 3D-QSAR models (CoMFA_ES and CoMSIA_EA) revealed various contour maps for understanding the essential features of structure-activity relationships of these molecules. The conventional hydrogen bond interactions with some key residues such as ARG118, GLU227, and ARG371 significantly made the 5-benzylidenethiazolinone moiety of the molecules to be more stable in both SA-cavity and 430-loop cavity of the pH1N1 neuraminidase from the docking studies. Six (6) **molecules (9, 10, 11, 17, 22, and 31)** with relatively high inhibitory activities, docking scores, and ADMET properties were identified as the possible lead molecules that can be utilized as templates for the in-silico design of novel candidates for anti-influenza therapy. Thus, the outcome of this study overlaid a solid foundation for the in-silico design and theoretical exploration of novel neuraminidase inhibitors with improved potency.

## Declarations

### Author contribution statement

Mustapha Abdullahi: Conceived and designed the experiments; Performed the experiments; Analyzed and interpreted the data; Contributed reagents, materials, analysis tools or data; Wrote the paper.

Adamu Uzairu, Gideon Adamu Shallangwa: Conceived and designed the experiments; Analyzed and interpreted the data.

Paul Andrew Mamza: Analyzed and interpreted the data.

Muhammad Tukur Ibrahim: Conceived and designed the experiments; Contributed reagents, materials, analysis tools or data.

### Funding statement

This research did not receive any specific grant from funding agencies in the public, commercial, or not-for-profit sectors.

### Data availability statement

Data included in article/supplementary material/referenced in article.

### Declaration of interests statement

The authors declare no conflict of interest.

### Additional information

No additional information is available for this paper.
